The article "Stress-mediated Sin3B activation leads to negative regulation of subset of p53 target genes" was retracted in 2024. Reasons: duplicated images; overlap with earlier publications; concerns about the images.

# Stress-mediated Sin3B activation leads to negative regulation of subset of p53 target genes

**DOI:** 10.1042/BSR20150122

**Published:** 2015-08-07

**Authors:** Rama Kadamb, Shilpi Mittal, Nidhi Bansal, Daman Saluja

**Affiliations:** * Dr. B. R. Ambedkar Center for Biomedical Research, University of Delhi, Delhi-110007, India

**Keywords:** gene regulation and bleomycin-induced stress, genotoxic stress, p53, Sin3B, Sin3–histone deacetylase (HDAC) complex, transrepression

## Abstract

The multiprotein SWI-independent 3 (Sin3)–HDAC (histone deacetylase) corepressor complex mediates gene repression through its interaction with DNA-binding factors and recruitment of chromatin-modifying proteins on to the promoters of target gene. Previously, an increased expression of Sin3B and tumour suppressor protein, p53 has been established upon adriamycin treatment. We, now provide evidence that Sin3B expression is significantly up-regulated under variety of stress conditions and this response is not stress-type specific. We observed that Sin3B expression is significantly up-regulated both at transcript and at protein level upon DNA damage induced by bleomycin drug, a radiomimetic agent. This increase in Sin3B expression upon stress is found to be p53-dependent and is associated with enhanced interaction of Sin3B with Ser^15^ phosphorylated p53. Binding of Sin3–HDAC repressor complex on to the promoters of p53 target genes influences gene regulation by altering histone modifications (H3K9me3 and H3K27me3) at target genes. Furthermore, knockdown of Sin3B by shRNA severely compromises p53-mediated gene repression under stress conditions. Taken together, these results suggest that stress-induced Sin3B activation is p53-dependent and is essential for p53-mediated repression of its selective target genes. The present study has an implication in understanding the transrepression mechanism of p53 under DNA damaging conditions.

## Abstract (precis)

Sin3B expression and its interaction with phosphorylated p53 increases under stress conditions. Recruitment of Sin3B by p53 at its target gene promoters is essential for the maintenance of inhibitory chromatin environment by inducing epigenetic modifications that brings about their target gene repression.

## INTRODUCTION

Gene regulation in eukaryotes is achieved through fine tuning of activator and repressor complexes that mediate relaxed and condensed chromatin state respectively. In general, two counteracting enzymes control the gene expression primarily: histone acetyltransferases (HATs) that add acetyl groups to the histone moieties and thus mediate gene activation; and the histone deacetylases (HDACs) which deacetylate histone proteins and thus contribute to gene repression [1]. These enzymes do not work individually, instead, they are recruited to the promoters of genes as multi-subunit protein complexes where other proteins function as chromatin remodellers and recruit additional cofactors or perform unknown functions [2]. Sin3, a negative regulator of gene transcription, is a component of HDAC co-repressor complex that is known to be involved in scaffolding of genome [3]. Like HDACs, Sin3 has no DNA-binding domain and interacts with various transcription factors through Sin3 interaction domain (SID) and thereby gets recruited on to the promoters of target genes [1,3,4]. Once recruited to the promoters, Sin3 executes gene repression by altering chromatin state through associated HDACs, such as Rpd3 (reduced potasium deficiency 3) in yeast and HDAC1 and HDAC2 in mammals [5,6].

In mammals, Sin3 has two paralogues; Sin3A and Sin3B which are known to perform varied functions under different cellular conditions [4,7]. Knockout studies in mice demonstrate distinct functions and differential requirement of the two isoforms during development. Loss of Sin3A is lethal during the early stages of development in mice and is required for T-cell development and maintenance of sarcomere structure [8,9]. In contrast, Sin3B is needed at later stages of development and is required for skeletal development and cell-cycle progression [10]. However, overlapping functions between these two paralogues cannot be ruled out as Sin3A is found to perform compensatory functions in the absence of Sin3B suggesting that there can be various complexes present in cell with different combinations of Sin3A/Sin3B [11–13]. Sin3 has recently been discovered to be involved in various cellular functions ranging from T-cell development, cell-cycle progression, differentiation, senescence, protein stabilization, energy metabolism and cell survival [4,8,9,12,14–20]. Apart from the above mentioned functions, role of Sin3 under DNA damage conditions has previously been studied in *Saccharomyces cerevisiae* where it mediates non-homologous end joining DNA repair [21]. However, the involvement of Sin3 under stress conditions is not well studied in higher organisms which prompted us to study the regulation of Sin3 in humans upon bleomycin treatment, a radiomimetic drug that causes double strand breakage [22,23]. Sin3 interacts with expanding array of DNA-binding transcription factors and our previous study affirmed interaction of Sin3B with p53, a stress-related protein [14,24–27]. p53 is exemplified as the ‘guardian of genome’ which gets rapidly activated upon exposure of cells to various stress signals [28,29]. p53 is a sequence-specific transcription factor that can either transactivate or transrepress various genes in a context-dependent manner [30]. The mechanism of p53-mediated gene activation and its role in regulation of damage/stress response pathways is well established [29,30]. However, the mechanism underlying p53-mediated transcriptional repression remains elusive. Previously, Sin3 has been demonstrated to play an imperative role in p53-mediated gene regulation [14,26]. Nevertheless, it is believed that different stress signals can lead to different, as well as independent pathways for p53 activation, which in turn can mediate different responses [31]. In the present study, we looked into the insight of mechanism of Sin3B activation and p53-mediated negative gene regulation under bleomycin-induced DNA damaging conditions. The present study shows that under bleomycin-induced stress, expression of Sin3B gets up-regulated and it gets recruited by p53 at its target promoters. Knockdown of Sin3B leads to impaired negative regulation of p53 target genes and thus exemplifies Sin3B as a critical player in down-regulation of p53 subset target genes.

## MATERIALS AND METHODS

### Cell culture and establishment of stably transfected cell lines

HCT116 (human colorectal carcinoma), KB (head and neck squamous carcinoma), A549 (human lung carcinoma), Saos2 (osteosarcoma) and H1299 (non small cell lung carcinoma) cell lines were cultured at 37°C in 5% CO_2_ humidified atmosphere. Cells were grown in high glucose Dulbecco modified Eagle's medium (DMEM; Sigma; Pan Biotech) supplemented with 10% FBS (Gibco) and penicillin (60 units/ml) and streptomycin (50 μg/ml). For transfection, HCT116 cells were seeded into six-well tissue culture plates and transfected with 1 μg of control/Sin3B shRNA plasmid (Santa Cruz Biotechnology) using plasmid transfection reagent according to manufacturer's protocol (Santa Cruz Biotechnology). Forty-eight hours after transfection, the positive clones were selected by growing cells in puromycin containing medium (ant-pr-1, Invivogen). KB, A549 and Saos2 cell lines were procured from National Center for Cell Sciences (NCCS) and HCT116 (wild-type and null for p53) and H1299 cell lines were provided as a kind gift from Dr Bert Vogelstein from John Hopkins University and Dr Sanjeev Das from National Institute of Immunology respectively.

### Cell treatment

Sub-confluent cultures were treated with different stress-inducing agents: cells were incubated with 400 μg/ml and 20 ng/ml of bleomycin and colchicine respectively, for indicated time points. For γ radiation treatment, cells at a confluency of 70%–80% were irradiated with γ radiation source (^60^Co; Eldorad78) in Hank's balanced salt solution (HBSS) and, after treatment, the cells were incubated at 37°C for 1 and 4 h respectively.

### Western blotting

Cells cultured in T25 cm^2^ flasks were subjected to different drug treatments for desired time intervals and harvested for analysing protein expression. Cell lysates were prepared by re-suspending the cells in RIPA (radioimmunoprecipitation assay) buffer for 45 min at 4°C. The soluble protein fractions were collected by centrifugation at 15 *777 **g***. Total protein was estimated using BCA protein estimation kit (Bangalore Genei) and equal amount of proteins (30 μg) were resolved on SDS/PAGE (either 8% or 10% gel) and transferred on to immunoblot- PVDF membranes (Santa Cruz Biotechnology). Following blocking with 5% BSA for 1 h at room temperature and washing with PBS with Tween 20 (PBST), the PVDF membranes were incubated overnight at 4°C in primary antibody (1:1000) diluted in PBST containing 1% BSA. Membranes were subsequently incubated with secondary antibodies conjugated with horseradish peroxidase (1:5000) for 1 h at room temperature. The blots were probed with the enhanced chemiluminescence (ECL) western blot detection system (Biogene) according to manufacturer's instructions.

### Co-immunoprecipitation

Sub-confluent cultures of untreated and bleomycin-treated cells were harvested and lysed in RIPA buffer (buffer composition as given in the Supplementary Table S1) supplemented with protease inhibitor cocktail (Sigma–Aldrich). Equal amount of protein (1.5 mg) from each sample was immunoprecipitated with 1 μg of desired antibody. For collection of the immunoprecipitates, 30 μl of protein A/G agarose beads were added to each tube and the samples were incubated for 2–3 h at 4°C on rotation. Each immunoprecipitate was washed thrice in RIPA buffer and eluted with 2× loading dye, fractionated on 8% SDS/PAGE and transferred overnight on to immuno-blot PVDF membrane (Santa Cruz Biotechnology). Immunodetection was done with anti-Sin3B antibody, p53 and phospho Ser^15^-p53 at a dilution of 1:1000 for Figures 3(A) and 3(B) respectively. Ten percent of the input was saved as a positive control from the total lysate.

### RNA purification, cDNA synthesis and qPCR

Untreated/control and bleomycin-treated cells were processed for RNA purification using RNeasy kit (Qiagen) according to manufacturer's instructions. One μg of RNA was used for cDNA synthesis using Verso cDNA kit (Thermo Scientific) according to the manufacturer's protocol. Semi-quantitative and quantitative real-time PCR (qPCR) reactions were carried out using gene specific primers. Real time gene expression analysis was carried out using MESA Green qPCR Mastermix plus for SYBR assay (Eurogenetec) on Applied Biosystems 7300 RT-PCR system and data were collected and exported with SDS 2.2.2 version. Relative expression was calculated using 2^−ΔΔC_t_^ method and 18S rRNA was used as an endogenous control. Sequence of primer pairs used for semi-quantitative and real-time PCR are listed in Supplementary Table S2.

### Cell-cycle analysis

To prepare cells for FACS analysis, 1×10^6^ (control and treated) cells were washed with 1× PBS, resuspended in 0.5 ml of 1× PBS and incubated with 10 μl of RNase A (10 mg/ml) at 37°C in a water bath for 30 min, followed by addition of 4 μg/ml of Propidium Iodide in dark on ice. Stained cells were analysed on Becton Dickinson FACScan machine and the data were analysed with either CELLQuest Pro or FlowJo software.

### ChIP (chromatin-immunoprecipitation)

HCT116 cells were treated with bleomycin drug prior to formaldehyde fixation. Formaldehyde fixed cells lysed in 0.1% SDS lysis buffer were sonicated (20 cycles of 30-s pulse with 1-min interval) at 90% power using Bioruptor sonicator (Diagenode). Samples were centrifuged for 10 min at 18516 ***g*** at 4°C and were diluted ten times with dilution buffer except for the input sample. The diluted supernatants were collected and pre-cleared with protein A/G Agarose beads containing 1 mg/ml salmon sperm DNA for 3–4 h at 4°C with agitation. Samples were spun down at 7012 ***g*** for 5 min at 4°C and incubated overnight with specific antibodies. Samples were incubated with 30 μl of pre-blocked beads (protein A/G agarose/salmon sperm DNA) for 3 h, spun at 986 ***g*** at 4°C for 3 min and washed sequentially with the following buffers at 4°C: once with 0.1% SDS lysis buffer, twice with low salt-wash buffer, twice with high salt-wash buffer, twice with LiCl wash buffer and twice with TE buffer. For de-cross-linking and PCR, samples were eluted twice with 100 μl of elution buffer, vortexed briefly and incubated at room temperature for 15 min with rotation. Eluates were pooled (200 μl) and 8 μl of 5 M NaCl added. De-cross-linking was performed at 65°C for 6 h to overnight. Following elution, samples were treated with 4 μl of 0.5 M EDTA, 4 μl of 1 M Tris, pH 6.8, 2 μl of 10 mg/ml proteinase K, 2 μl of 10 mg/ml RNAase A and incubated for 3 h at 45°C. DNA from eluted samples was recovered with PureLink PCR purification Kit (Invitrogen). PCR and quantitative real time PCR were performed using gene-specific primers for promoter regions. Composition of the buffers and primer pairs used are given in Supplementary Tables S1 and S3.

### Statistical analysis

Student's *t*-test was used to evaluate the significance of the differences between control and drug-treated samples in all pertinent experiments; a *P*-values<0.05 and 0.01 was considered significant and highly significant respectively.

## RESULTS

### Sin3B expression is induced upon different cellular stress conditions and is not cell-type specific

Cell lines of different origins were subjected to genotoxic (bleomycin and γ-radiation) and non-genotoxic stress (colchicine) to study their effect on the expression of human Sin3B and stress-related protein, p53. Initially, the dose of bleomycin which can induce cellular stress and thus elicit p53 activation was standardized. It was found that 400 μg/ml of bleomycin drug is sufficient to activate p53 levels and lead to arrest of cells in the G_2_-phase of the cell cycle (Supplementary Figures S1A and S1B). Western blot analysis of lysates from untreated and treated cells depicted time-dependent increase in the expression of Sin3B and p53 upon bleomycin drug treatment as compared with control cells (Figure 1A, left panel). The expression of both Sin3B and p53 showed significant increase at protein level within 20 min after bleomycin treatment and these high levels of protein expression were maintained up to 24 h post drug treatment. The expression levels of p53 and Sin3B at 24 h after bleomycin treatment was approximately 5- and 2.5-fold higher respectively as compared with controls (Supplementary Figure S1C). This increase in expression of Sin3B was not isoform specific as we observed similar increase in the levels of another Sin3 isoform, i.e. Sin3A in bleomycin-treated cells (Supplementary Figure S1D). Similarly, exposure of cells to 5 Gy of γ-radiation dose lead to enhanced Sin3B expression at 1 and 4 h with a concomitant increase in the p53 levels (Figure 1B).

**Figure 1:** Expression of Sin3B increases under conditions of cellular stress in a p53-dependent manner HCT116 wild-type (HCT116 p53^+/+^) cells were treated with different stress inducers that are known to elicit p53 activation and response. (**A**) Cells were subjected to bleomycin (radiomimetic agent) and colchicine (mitotic poison) drug treatment at 400 μg/ml and 20 ng/ml dose respectively, at indicated time points. (**B**) KB cells were subjected to γ-radiation at a dose of 5 Gy and incubated for 1 and 4 h in HBSS. (**C**)Western blots showing expression of Sin3B and p53 protein in KB and A549 cell lines. (**D**) Western blot analysis showing no effect on the expression of Sin3B in p53 null cells (HCT116 p53^−/−^). Following different drug treatments, the expression of p53 and Sin3B were checked by performing western blot analysis using specific antibodies. For all the experiments, β-actin was used as endogenous control.

Under conditions of non-genotoxic stress, induced by colchicine (mitotic poison), we observed that expression of Sin3B began to increase within 30 min after treatment with colchicine drug at a concentration of 20 ng/ml and time-dependent increase was observed till 16 h of drug incubation (Figure 1A, right panel). In concordance to published reports, we also observed that exposure of cells to different kinds of stress stimuli was accompanied by an increase in p53 protein level. We also demonstrate that increased expression of Sin3B, upon bleomycin treatment, is not cell-type specific as cell lines of different origins (head and neck squamous carcinoma and non-small cell lung carcinoma) treated with bleomycin showed similar increase in Sin3B expression (Figure 1C).

Further, to gain insight into the role of p53 in Sin3B regulation, p53 null cells were subjected to similar conditions of stress and analysed for protein expression. Importantly, p53 null cells did not show any significant increase in Sin3B expression upon bleomycin drug treatment neither at protein nor at transcript levels (Figure 1D; Supplementary Figure S2). These results evinced that increase in Sin3B expression level upon stress conditions is a general phenomenon that can occur in a variety of cell type regardless of the stimulus types that initiate this process and p53 is required for Sin3B activation.

### Increased Sin3B expression is due to increased transcript level and post-translational stabilization

To ascertain whether increase in Sin3B protein upon cellular stress is a result of increased transcription, total RNA from control and bleomycin-treated samples were isolated and reverse transcribed. Semi-quantitative and qPCR indicated a significant increase in the levels of Sin3B transcript; however, no changes were observed for p53 transcript levels upon bleomycin treatment (Figures 2A and 2B). To rule out the possibility of ineffective drug treatment for insignificant changes in p53 expression, transcript levels of p21 gene were also analysed simultaneously. p21 is a well-known p53 target gene which gets up-regulated under variety of stress conditions [29]. We observed significant increase in p21 transcript levels following bleomycin treatment, confirming that the drug treatment is indeed effective (Supplementary Figure S3). In the current study, no significant changes in the p53 mRNA levels (Figure 2A) are consistent with previous studies that suggest p53 expression is typically enhanced at post-translational level under stress conditions [32]. In contrast, a significant increase was observed for Sin3B mRNA levels within 20 min of bleomycin drug treatment that further increased up to 4-fold in a time-dependent manner (Figure 2B).

**Figure 2:** Human Sin3B transcript levels are increased upon bleomycin treatment Total RNA was isolated and reverse transcribed at various time point as indicated in the figure. The cDNA (control and treated samples) was used as a template for semi-quantitative PCR as well as for qPCR using gene-specific primers. (**A** and **B**) represents the expression of p53 and Sin3B transcripts respectively as detected by qPCR (upper panels) and semi-quantitative PCR (lower panels) in HCT116 cell line after bleomycin treatment at different time points. Relative expression levels were calculated by taking transcript level in untreated cells as one. The C_t_ value for each gene was normalized with 18S rRNA which was used as an endogenous control. Error bar shows S.D. and the plots have been plotted with ± S.E.M. *P<0.05 and **P<0.01. For semi-quantitative PCR, p53 and Sin3B were amplified for 28 and 30 cycles respectively. The results are representative of three independent experiments. (**C**) Western blot analysis of cell lysates from bleomycin-untreated and -treated samples at various time points as indicated in the figure for checking the expression levels of Sin3B and RNF220, a ubiquitin ligase. β-actin was used a protein loading control.

We next checked whether augmentation of Sin3B protein upon stress was a result of increased translational product alone (due to increase in mRNA for Sin3B) or post-translational stabilization has any role to play in increasing Sin3B protein levels. Previously, RNF220 (ring finger protein 220) protein has been identified as a novel ubiquitin ligase of Sin3B [33]. We, therefore, compared the expression levels of RNF220 protein along with Sin3B protein under similar stress conditions. Western blot analysis showed that expression of RNF220 decreased as a function of time of bleomycin treatment with a concomitant increase in the expression of Sin3B protein (Figure 2C). Thus, our results suggest that increased expression of Sin3B at protein level is a cumulative effect of increased transcript synthesis and increased stabilization due to decreased RNF220 expression upon bleomycin treatment.

### Increased association of human Sin3B with p53 phosphorylated at Ser^15^

Human p53 is known to undergo several post-translational modifications (PTMs) through activation of several kinases. Using co-immunoprecipitation and yeast two-hybrid studies, we earlier reported that p53 directly interacts with Sin3B under normal conditions without any increase in association between the two proteins under adriamycin-induced stress conditions [14]. Out of the many types of phosphorylation, p53 phosphorylation on Ser^15^ residues occurs following DNA damage induced by γ-radiation and several chemotherapeutics agents [34–36]. To study the effect of PTM of p53 on its interaction with Sin3B, under stress conditions, co-immunoprecipitation assays were performed. Initially, expression of Ser^15^ phosphorylated p53 was investigated in control and 24 h drug-treated HCT116 cells. Western blot analysis showed that levels of Ser^15^ phosphorylated at p53 residues increased after treatment of cells with bleomycin (Supplementary Figure S4). Following confirmation of p53 modification at Ser^15^ residues after bleomycin treatment, protein lysates from untreated and drug-treated cells were immunoprecipitated using p53 and phospho Ser^15^-p53 antibody followed by immunoblotting with Sin3B-specific antibody. Co-immunoprecipitation assay with total pool of p53 showed no increased association of Sin3B under bleomycin-induced stress; however, immunoprecipitation of the complex with phospho Ser^15^-p53 antibody followed by detection with anti-Sin3B antibody showed enhanced interaction between Ser^15^ phosphorylated p53 and Sin3B (Figure 3A).

**Figure 3:** Increased physical association occur between Sin3B and phosphorylated pool of p53 (Ser^15^) in bleomycin-treated cells (**A**) Cell lysates from untreated and 24 h bleomycin drug-treated cells were immunoprecipitated (IP) with antibodies specific for p53 and phospho Ser^15^-p53 followed by immunoblotting (IB) with antibody specific to Sin3B. (**B**) Reciprocal co-immunoprecipitation in HCT116 wild-type cells using anti-Sin3B antibody for immunoprecipitation of the immune complex and anti-p53 antibody for immunodetection. Input corresponding to 10% of the total cell lysate was used as a positive control whereas mouse and rabbit IgG were used as negative controls.

In contrast, no significant band was observed in the isotype (mock) lane that confirmed the specificity of interaction. Reciprocal immunoprecipitation-western experiments using anti-Sin3B antibody for immunoprecipitation of the complex and anti-p53 antibody for immunodetection demonstrated that Sin3B could also co-immunoprecipitate p53 under similar conditions. This, further, affirmed the specific interaction between these two proteins (Figure 3B).

### Sin3–HDAC complex docks on to the promoter of subset of p53 target genes

To decipher the functional significance of human p53–Sin3B interaction and to understand the role played by Sin3B in p53-mediated gene regulation upon bleomycin treatment, the recruitment of human Sin3B on to the five selected p53 responsive promoters was investigated. Whereas Sin3 has been shown to stabilize p53 for mediating its transrepression functions [20,26], there has been no comprehensive study regarding the role of Sin3B in p53-mediated negative gene regulation under bleomycin-induced DNA damaging situations.

To study the recruitment of Sin3B on to p53 target promoters, ChIP assays were performed with cellular extracts from untreated and 24-h bleomycin-treated HCT116 cells, using promoter-specific primers designed across the p53-response element (RE). In the initial screening phase, we observed significant enrichment of human Sin3B on five out of eight p53-target promoters, viz. *MAD1* (mitotic arrest deficient-like 1), *HSPA8* (heat-shock 70 kDa protein 8), *CRYZ* (crystallin, zeta), *ANLN* (anillin) and *CDC25c* (cell division cycle 25C; result not shown) and hence, focused at these five promoters only for a detailed dissection of the involvement of Sin3B in p53-mediated gene repression. Using specific antibodies against p53, Sin3B and HDAC1, substantial recruitment of these three proteins at the region spanning the p53 REs were observed for the five p53 target genes under both normal and stressed conditions. The strength of the specific binding of antibodies was evident when compared with isotype control (Figure 4A).

**Figure 4:** Recruitment of p53–Sin3B–HDAC1 occurs on subset of p53 target genes ChIP assays were performed in HCT116 cells in untreated and cells treated with bleomycin for 24 h. Equal amounts of cross-linked chromatin were pre-cleared and incubated with 1μg of antibody for anti-p53, anti-Sin3B, anti-HDAC1 as indicated above each lane. Following DNA precipitation, samples were analysed by PCR using specific primers for *HSPA8*, *MAD1*, *CRYZ, CDC25c* and *ANLN.* Input corresponding to 10% of the total chromatin used as positive control for each immunoprecipitation reaction and IgG was used as isotype control. * Indicates primer dimers. (**B**) For RT-PCR assays, ChIP DNA recovered from each immunoprecipitation using specific antibodies for p53, Sin3B and HDAC1 was used as a template and amplified using gene-specific primers with SYBR green dye on ABI-7300 system. Amplification in the mock (isotype) was used as control. Percent input was calculated for enrichment of DNA on to the respective target promoters in bleomycin control and bleomycin-treated conditions.

qPCR assay was performed to further investigate that whether any enrichment occurs for p53, Sin3B and HDAC1 at the p53 target promoters in the presence and absence of bleomycin drug treatment. For this, ChIP DNA obtained after immunoprecipitation with specific antibody (Figure 4B) from both untreated and drug-treated cells was used as a template and amplified using gene-specific primers. Our qPCR results were in agreement with ChIP PCR results that showed no significant changes in the recruitment of p53, Sin3B and HDAC1 at selective p53 target promoters in bleomycin-treated cells as compared with untreated cells (Figure 4B).

### Negative regulation of subset of p53 target genes is Sin3B dependent

To further validate the role of Sin3B in stress-induced p53-mediated gene repression of its target genes, we transfected the HCT116 cells with Sin3B shRNA to knockdown Sin3B (KDB) expression. Cells transfected with shRNA showed significant reduction in the expression of Sin3B as compared with untransfected cells both at protein and at RNA level (Figure 5A). Densitometric analysis revealed that Sin3B shRNA treatment resulted in approximately 80% reduction in the expression of Sin3B in transfected cells as compared with untransfected cells.

**Figure 5:** Knockdown of Sin3B inhibits p53-mediated repression of its target genes (**A**) HCT116 cells were transfected with control and Sin3B shRNA and the expression of Sin3B was analysed in control and bleomycin-treated transfected cells through western blotting (left panel) and semi-quantitative PCR (right panel). (**B**) Cell cycle profile of HCT116 cell line in control shRNA (upper panel) and upon transfection with Sin3B shRNA (lower panel) in untreated and drug-treated cells. (**C**) Expression levels of p53 target genes were analysed in control and Sin3B shRNA transfected cells under both untreated and bleomycin-treated conditions. Relative expression levels for each gene were calculated by considering transcript levels of genes in untreated conditions as one. 18s rRNA was used as endogenous control. Error bar shows S.D. and the plots have been plotted with ± S.E.M. *P<0.05 and **P<0.01. Abbreviations: BC, bleomycin control; BT, bleomycin treated.

Knockdown of Sin3B in *Drosophila* S2 cells is known to cause arrest of cells in the G_2_-phase of the cell cycle [17]. Therefore, we also investigated whether knockdown of Sin3B in HCT116 cell line causes any cell-cycle perturbation. Using Propidium Iodide staining, cell cycle profile of untransfected and Sin3B shRNA transfected cells were analysed under normal and bleomycin-induced DNA damage conditions. Cell cycle analysis revealed that significant fraction of cells entered G_2_-phase of cell cycle in cells ablated for Sin3B as compared with untransfected cells upon bleomycin treatment. However, no significant changes in the cell cycle patterns were observed between untransfected and Sin3B transfected cells under normal cycling conditions/without drug treatment (Figure 5B). We next checked for the effect of Sin3B knockdown on the expression of p53 target genes following bleomycin drug treatment. We observed significant derepression of the p53 target genes in the cells transfected with Sin3B shRNA upon bleomycin treatment. In contrast, untransfected cells showed significant repression of the same target genes under similar conditions (Figure 5C).

Thus, our results highlight the importance of Sin3B in negatively regulating p53 gene repression under bleomycin-induced stress conditions.

### Induction of epigenetic modifications on promoters of p53 target genes

Sin3B–HDAC complex is associated with enzymes involved in histone methylation and such PTMs at histones play critical role in gene regulation [10,37]. We, therefore, tested whether bleomycin-mediated stress alters the methylation marks on histones at promoters of p53 target genes. To better understand this phenomenon, HCT116 wild-type cells were treated with bleomycin and the endogenous promoter occupancy was examined on formaldehyde cross-linked chromatin by using specific antibodies for H3K4me3 as activation mark and H3K9me3/H3K27me3 as repression marks. To monitor the specificity of reaction, IgG was used as an isotype control. ChIP assay revealed that exposure of cells to bleomycin drug did not cause any change in the enrichment of H3K4me3 except for *MAD1* gene (Figure 6). However, significant increase in hypermethylation of H3K9me3/H3K27me3, repression marks, was observed after bleomycin drug treatment. At the promoter of *HSPA8* gene, we observed increased hypermethylation of H3K9me3 residues with no significant change in trimethylation of His^3^ at Lys^27^ residues. In contrast, *CDC25c* promoter showed increased hypermethylation for H3K27me3 residue without any significant changes for the other repression mark, i.e. H3K9me3. However, at *MAD1, CRYZ* and *ANLN* promoter sites, we observed an increased hypermethylation of both the repression marks, i.e. H3K9me3 and H3K27me3 (Figure 6). These observations suggested that differential hypermethylation of histones occur following bleomycin treatment and such changes are responsible for bleomycin-mediated p53 gene repression of its target genes.

**Figure 6:** Epigenetic modifications occur at the promoters of p53 target genes upon bleomycin treatment HCT116 wild-type untreated and 24 h bleomycin drug-treated cells were harvested for ChIP assay. Equal amounts of cross-linked chromatin were pre-cleared and incubated with antibodies methylated at different residues of His^3^ as indicated in the figure. Following DNA precipitation, samples were analysed by qPCR using specific primers for *HSPA8*, *MAD1*, *CRYZ, CDC25c* and *ANLN* promoters. Error bar shows standard deviation and the plots have been plotted with ± S.E.M. *P<0.05 and **P<0.01. Percent input was calculated for enrichment of DNA on to the respective target promoters in bleomycin control and bleomycin treated conditions.

## DISCUSSION

Several lines of evidence suggest that p53 modulates gene expression under diverse environmental, genotoxic and developmental stimuli by different mechanisms of transrepression [14,38,39]. Furthermore, the mechanism of transrepression being context-dependent, interaction and cross-talk between these pathways cannot be ruled out. It is also well established that several cellular insults/stimuli induce p53 expression [32]. However, the regulation/response of Sin3B under such scenario is still not clear. We, now provide evidence that expression of Sin3B increases in p53-dependent manner under variety of stress conditions. Though, increase in Sin3B expression was also observed upon Rat Sarcoma (Ras) oncogene activation and adriamycin treatment to cells [14,40]; the mechanism of Sin3 up-regulation is still far from clear. Previously, RNF220, a ubiquitin ligase, has been shown to associate with Sin3B and promotes its proteasomal degradation [33]. In the present study, we found that expression of RNF220 decreased with a concomitant increase in Sin3B expression upon bleomycin treatment. At the RNA level, our qPCR results indicate significant increase in the Sin3B transcripts in a time-dependent manner following bleomycin treatment. These observations suggest that increased Sin3B expression at protein level is a cumulative effect of both increased transcript synthesis and post-translational stabilization by RNF220. In contrast, the expression of p53 increased at protein level only with no significant change in transcript level upon bleomycin treatment. Thus, our observation further supports the fact that p53 is post-translationally stabilized under stress [32]. Interestingly, we did not find stress-induced expression of Sin3B in p53 null cells neither at protein nor at transcript levels (Figure 1D; Supplementary Figure S4). These findings, though, imply that increase in Sin3B expression might be regulated through p53 (directly or indirectly); the mechanism for gene regulation cannot be explained as of this writing as promoter of Sin3B is yet not identified. We further looked into the Sin3B gene in search for any consensus p53-binding site using TRANSFAC program. However, we did not find any p53-binding site upstream of the putative transcription start site of Sin3B gene. Thus, in future, due attention is required to study the transcriptional and post-translational regulation of Sin3B by p53, especially under the conditions of stress.

Our previous studies suggested that Sin3B interacts with N-terminal region of p53 under normal as well as stress conditions [14]. However, the interaction status between p53 and Sin3B does not change upon adriamycin drug treatment [14]. Like adriamycin, we found that bleomycin also does not cause any change in the interaction status of Sin3B with total pool of p53. Interestingly, in the present study, we observed that, association of Sin3B is increased with Ser^15^ phosphorylated p53 under stress conditions. In response to DNA damage, Ser^15^ and Ser^20^ residues of p53 primarily get phosphorylated and blocks its interaction with mouse double minute 2 (MDM2), a negative regulator of p53 [41–43]. Ser^15^ phosphorylation has been shown to enhance the interaction of p53 with various transcription factors. Phosphorylation of p53 at Ser^15^ residues is reported to result in increased association of p53 with CREB (cAMP-RE-binding protein) under DNA damage conditions. In fact, phosphorylation of the p53 at N-terminus is shown to be involved in controlling protein interaction, regulating transcription of downstream genes and it may also contribute in determining the response of cells to DNA damage [44]. Thus, our results are in concordance with published reports that propose phosphorylation of p53 in mediating increased interaction with other proteins [44]. Although, it remains unclear that whether this increase in p53 Ser^15^–Sin3B interaction represents an increase in binding affinity or binding stoichiometry and thus in future needs to be explored in detail.

In order to check whether the association of p53 with Sin3B results in modulating the expression of downstream target genes, recruitment of Sin3B–HDAC1 was analysed on to selective promoters of p53 target genes. A consistent recruitment of p53–Sin3B–HDAC1 on to the promoters of p53 repressed genes was observed both before and after DNA damaging conditions. Ceribelli and co-workers showed that for genes, like ataxia telangiectasia and Rad3-related protein (ATR), casitas B-lineage lymphoma (CBL), clusterin (CLU), HMG-coA reductase degradation protien 1 (HRD1) and replication factor C (RFC4), the levels of p53 bound to the target promoters do not seem to be affected following adriamycin treatment as compared with untreated cells [45]. Further, p53 and nuclear transcription factor-Y (NF-Y) transcriptional factors are known to be recruited/associated on to the promoters of cyclin B2, *CDC25c* and cyclin dependent protein kinase 2 (*CDC2*) genes before and after DNA damage [14,45–47]. Thus, our results are in agreement with literature that suggests binding of p53 under normal and cellular stress conditions. p53 is a sequence-specific transcription factor that can bind to several target promoters but in few cases it has been suggested that mere binding of a transcription factor to a specific genomic sequence does not necessarily imply direct transcriptional regulation. Therefore, we also checked the expression of p53 target genes in HCT116 (p53^+/+^) cell line to observe the downstream effect of p53–Sin3B–HDAC1 recruitment on to the target promoters upon bleomycin treatment. We found that although we did not observe any difference in the enrichment of p53–Sin3B–HDAC1 on to the promoters but significant down regulation of the same target genes was observed in bleomycin-treated cells as compared with control cells.

Since, we observed the up-regulation of Sin3B following exposure of cells to any kind of stress stimuli and recruitment of Sin3B on to p53 target promoters, therefore we performed knockdown assays to find out the role of Sin3B in modulation of p53 target genes. Our data in cells ablated for Sin3B using Sin3B shRNA showed highly significant derepression of subset of p53 target genes as compared with untransfected cells. The derepression of p53 target genes was seen only under bleomycin-induced DNA damaging conditions. Untransfected and Sin3B shRNA transfected cells showed no significant changes under the normal cell cycling conditions. However, following Sin3B shRNA treatment we could not observe complete derepression of the p53 target genes. This lack of complete derepression after transfection of Sin3B shRNA could be attributed to the fact that Sin3 gene has two paralogues, i.e. Sin3A and Sin3B. Both paralogues show structural similarity with each other and regulate unique, as well as overlapping subset of target genes [3,7,20,26,48,49]. It is believed that in the absence of Sin3B, the other isoform, namely Sin3A, can substitute for it and take over the function. Sin3A associates with transcription regulators like methyl CpG binding protein 2 (MeCP2) and silencing mediator of retinoic acid and thyroid hormone receptor (SMRT) whereas on the other hand Sin3B preferentially associates with MHC Class II Transactivator (CIITA) and major histocompatibility complex (MHC II) [50–52]. Previously, Sin3A isoform has been shown to be involved in negative regulation of microtubule-associated protein 4 (*MAP4*) and stathmin (*STMN1*) genes [20,26]. Studies by van Oevelen et al. [12] have shown that both the isoforms are required for the maintenance of sarcomere functions and deletion of any one of the paralogues cannot rescue the normal phenotype [3].

Interplay of DNA and histone modifications via histone methyl transferases are prerequisite for regulation of gene expression. Sin3 associates with RBP2 (retinol-binding protein 2) through SAP30 (Sin3-associated protein 30) and recruits histone methyltransferase Suv39H1 (suppressor of variegation 3–9 homologue 1) that results in trimethylation of hypoacetylated H3K9 and provides a binding platform for the chromodomain of HP1 (heterochromatin-binding protein 1) protein [10,37,53,54]. This tethering of Sin3B–RBP2–HP1 leads to chromatin compaction. The Sin3 core complex contains Sin3A/Sin3B, HDAC1/HDAC2, Sin3 associated protein 18 (SAP18), ING1/2 (inhibitor of growth protein 1/2) and retinoblastoma-associated proteins (RbAps) that serves as a scaffold for additional moieties with enzymatic functions, such as nucleosomal remodelling, *N*-acetylglucosamine transferase, DNA methylation and histone methylation [10,37]. In the present study, we observed that the mechanism of p53-mediated gene repression is via the recruitment of Sin3–HDAC complex-associated epigenetic modifications on to p53 target gene promoters. We suggest that differential hypermethylation in response to bleomycin-induced DNA damage for different p53 target genes are responsible for gene regulation. Interestingly, we observed increased hypermethylation of H3K4, a well-known activation marker on to MAD1 promoter along with H3K9 and H3K27 repression marks. Trimethylation of His^3^ at Lys^4^ residues predominantly acts in transcription up-regulation activities. However, Shi et al. [55] showed that trimethylated H3K4 recruits Sin3–HDAC complex through plant homeodomain (PHD) domain of ING 2, a subunit of Sin3–HDAC complex in response to DNA damage and brings about gene repression. Apart from methylation, role of other PTMs of histones and DNA in regulating the transcriptional activities of these genes cannot be ruled out.

In the present report, we investigated the mechanism of p53-mediated repression of target promoters, active in the regulation of heat-shock maintenance, cell cycle and cytoskeleton regulation under bleomycin-induced DNA damaging conditions. We came to the following conclusions: (i) Sin3B acts as a stress-related protein whose expression increases upon exposure to a variety of cellular stimuli; (ii) Interaction of Sin3B with p53 phosphorylated at Ser^15^ residues is enhanced under stress conditions; (iii) Presence of Sin3B is crucial for repression of selective p53 target genes under stress conditions. Based on all these observations, we propose that direct binding of p53 to its REs is associated with recruitment of Sin3–HDAC complex. However, in the absence of any external stimuli, this complex is unable to induce any chromatin modifications. On the other hand, once a cell is subjected to DNA damaging stimuli (such as bleomycin), the Sin3–HDAC complex can bring about the histone modifications on to the promoters of selective p53 target genes that mediates chromatin compaction resulting in gene repression.

## Abbreviations

ANLN: anillin
BC: bleomycin control
BT: bleomycin treated
CDC25c: cell division cycle 25C
CRYZ: crystallin, zeta
HDAC: histone deacetylase
HBSS: Hank's balanced salt solution
HP1: heterochromatin-binding protein 1
HSPA8: heat-shock 70 kDa protein 8
IP: immunoprecipitation
KDB: knockdown Sin3B
MAD1: mitotic arrest deficient-like 1
PBST: PBS with Tween 20
PTM: post-translational modification
qPCR: quantitative real-time PCR
RBP2: retinol-binding protein 2
RE: response element
RIPA: radioimmunoprecipitation assay
RNF220: ring finger protein 220
Rpd3: reduced potassium dependency
RT: real time
SAP: Sin3-associated protein
Sin3: SWI-independent
